The article "Long non-coding RNA TUG1 knockdown hinders the tumorigenesis of multiple myeloma by regulating the microRNA-34a-5p/NOTCH1 signaling pathway" was retracted in 2021. Reason: misconduct by an author.

# Long non-coding RNA TUG1 knockdown hinders the tumorigenesis of multiple myeloma by regulating the microRNA-34a-5p/NOTCH1 signaling pathway

**DOI:** 10.1515/biol-2020-0025

**Published:** 2020-06-09

**Authors:** Yongtian Zhang, Dandan Zhao, Shumei Li, Meng Xiao, Hongjing Zhou, Shuige Yang, Yunliang Hao, Shasha Dong

**Affiliations:** Department of Hematology, Ji’ning No. 1 People’s Hospital, Ji’ning, Shandong, China

**Keywords:** long non-coding RNA, TUG1, microRNA-34a-5p, NOTCH1, multiple myeloma

## Abstract

Multiple myeloma (MM) is a serious health issue in hematological malignancies. Long non-coding RNA taurine-upregulated gene 1 (TUG1) has been reported to be highly expressed in the plasma of MM patients. However, the functions of TUG1 in MM tumorigenesis along with related molecular basis are still undefined. In this study, increased TUG1 and decreased microRNA-34a-5p (miR-34a-5p) levels in MM tissues and cells were measured by the real-time quantitative polymerase reaction assay. The expression of relative proteins was determined by the Western blot assay. TUG1 knockdown suppressed cell viability, induced cell cycle arrest and cell apoptosis in MM cells, as shown by Cell Counting Kit-8 and flow cytometry assays. Bioinformatics analysis, luciferase reporter assay, and RNA pull-down assay indicated that miR-34a-5p was a target of TUG1 and directly bound to notch receptor 1 (NOTCH1), and TUG1 regulated the NOTCH1 expression by targeting miR-34a-5p. The functions of miR-34a-5p were abrogated by TUG1 upregulation. Moreover, TUG1 loss impeded MM xenograft tumor growth *in vivo* by upregulating miR-34a-5p and downregulating NOTCH1. Furthermore, TUG1 depletion inhibited the expression of Hes-1, Survivin, and Bcl-2 protein in MM cells and xenograft tumors. TUG1 knockdown inhibited MM tumorigenesis by regulating the miR-34a-5p/NOTCH1 signaling pathway *in vitro* and *in vivo*, deepening our understanding of the TUG1 function in MM.

## 1 Introduction

Multiple myeloma (MM), characterized by the infiltration and growth of malignant plasma cells in the bone marrow, accounts for about 10% of hematological malignancies [1,2]. It was estimated that approximately 159,985 new MM cases and 106,105 MM-related deaths occurred in 2018 worldwide [3]. Although considerable progress has been made in the management of MM, the prognosis for MM patients is still unsatisfactory with a median survival of around 6–7 years [2,4]. Increased understanding of the molecular pathogenesis of MM is crucial to improve the therapeutic outcomes for MM patients and reduce its detriment to patients.

Long non-coding RNAs (lncRNAs), a group of non-protein-coding transcripts greater than 200 nucleotides (nt) in length, have been well documented as crucial regulators in a wide range of biological processes including proliferation, cell cycle progression, and apoptosis [5,6]. Emerging evidence showed that lncRNAs played crucial roles in the development and progression of multiple types of tumors including MM [7,8]. lncRNA taurine-upregulated gene 1 (TUG1), located on chromosome 22q12.2 in humans, has been widely reported as an oncogenic factor with aberrant upregulation in many malignancies [9,10]. For instance, TUG1 knockdown weakened migratory, invasive, and proliferative abilities of renal cell carcinoma cells and promoted renal cell carcinoma cell apoptosis [11]. TUG1 loss suppressed cell proliferation, migration, invasion, and induced cell cycle arrest and cell apoptosis in laryngeal squamous cell carcinoma [12]. However, TUG1 has been found to be a tumor suppressor to hamper tumorigenesis in glioma and non-small-cell lung carcinoma [13,14]. Isin et al. pointed out that the TUG1 expression was markedly upregulated in the plasma of MM patients than that in the healthy control group [15]. However, little is known about the roles and molecular mechanisms of TUG1 in the tumorigenesis of MM.

The article "Long non-coding RNA TUG1 knockdown hinders the tumorigenesis of multiple myeloma by regulating the microRNA-34a-5p/NOTCH1 signaling pathway" was retracted in 2021. Reason: misconduct by an author.

MicroRNAs (miRNAs) are a class of short RNAs (approximately 21 nt) that have no or little protein-coding potential [16]. Mounting evidence manifested that miRNAs played a major role in various physiological and pathological processes by regulating the translation and stability of target mRNAs at the post-transcriptional levels [16,17]. Moreover, a growing body of literature supported the notion that miRNAs can exert anti-tumor or carcinogenic activity in MM [18]. lncRNAs have been proposed as competing endogenous RNAs (ceRNAs) of miRNAs to relieve the inhibition of gene expression caused by miRNAs [19,20].

In this study, the roles and miRNA targets of TUG1 in the tumorigenesis of MM together with the downstream regulatory pathways are further investigated in the MM cells and xenograft tumor models.

## 2 Materials and methods

### 2.1 Clinical samples

MM patients (26 males, 23 females; median age: 61.6 years old; international staging system stage 1: 8, stage 2: 21, and stage 3: 20) free from other diseases and healthy volunteers (10 males, 6 females; median age: 59.2 years old) were recruited from Ji’ning No. 1 People’s Hospital. Bone marrow samples were collected from these MM patients and healthy volunteers at the time of the diagnosis.


**Informed consent:** Informed consent has been obtained from all individuals included in this study.
**Ethical approval:** The research related to human use has been complied with all the relevant national regulations, institutional policies and in accordance with the tenets of the Helsinki Declaration, and has been approved by the Ethics Committee of Ji’ning No. 1 People’s Hospital.

The article "Long non-coding RNA TUG1 knockdown hinders the tumorigenesis of multiple myeloma by regulating the microRNA-34a-5p/NOTCH1 signaling pathway" was retracted in 2021. Reason: misconduct by an author.

### 2.2 Cell culture

Three MM cell lines (NCI-H929, MM.1S, and U266) were purchased from American Type Culture Collection (ATCC, Manassas, VA, USA). Normal plasma cells (nPCs) were sorted from bone marrow of healthy volunteers by the FACS Calibur flow cytometer cytometry (BD Biosciences, San Jose, CA, USA) via the following four surface markers: CD45-PB, CD56-PE, CD38-FITC, and CD19-PC7. Immunophenotype of nPCs was CD45+/dimCD38+CD19+CD56−. NCI-H929 cells were grown in the RPMI-1640 medium (Thermo Fisher Scientific, Waltham, MA, USA) supplemented with 2-mercaptoethanol (0.05 mM; Sigma-Aldrich, St Louis, MO, USA) and 10% fetal bovine serum (FBS; Thermo Fisher Scientific). MM.1S, U266 and nPCs cells were cultured in the RPMI-1640 medium (Thermo Fisher Scientific) containing 10% FBS. All the cells were maintained in a humidified air of 5% carbon dioxide (CO_2_) at 37°C.

### 2.3 Reagents and cell transfection

The TUG1 overexpression vector (TUG1) was obtained by cloning the sequence of TUG1 pcDNA3.1 (Genomeditech, Shanghai, China). Before transfection, NCI-H929 and U266 cells were seeded in a 12-well plate. Then, 0.2 μg of TUG1 was transfected in NCI-H929 and U266 cells (4 × 10^5^ cells/well, 80% confluency) with 0.5 μL of Lipofectamine 3000 reagent (Thermo Fisher Scientific). Furthermore, those oligonucleotides included three small interfering RNAs (siRNAs) targeting TUG1 (siTUG1-1, siTUG1-2, and siTUG1-3) and a scramble control (scrambled) (GenePharma, Shanghai, China); microRNA-34a-5p (miR-34a-5p) mimic and its negative control miR-NC (Thermo Fisher Scientific) were transfected into NCI-H929 and U266 cells using 0.6 μL of Lipofectamine 3000 transfection reagent (Thermo Fisher Scientific).

### 2.4 Real-time quantitative polymerase reaction assay

Extraction and purification of RNA were performed using the TRIzol reagent (Thermo Fisher Scientific) and RNase-free DNaseI (Thermo Fisher Scientific). RNA was quantified using a NanoDrop ND-1000 Spectrophotometer (NanoDrop, Wilmington, MA, USA), and its purity was detected using the A260/280 ratio. The miR-34a-5p level was measured using the TaqMan™ MicroRNA Reverse Transcription Kit and TaqMan™ MicroRNA Assay Kit (Thermo Fisher Scientific) with small nuclear RNA U6 as the internal reference. In brief, the transcription was conducted in a 10 μL reaction mixture, including polyadenylated RNA (100 ng), 5× PrimeScript buffer (2 μL), PrimeScript RT enzyme mix I (0.5 μL), RT primer mixture (1 μL), and RNase-free water. Whereafter, the total reaction mixture was incubated at 50°C for 15 min and 85°C for 5 s. For the quantitative analysis of TUG1 and notch receptor 1 (NOTCH1), RNA was reversely transcribed into cDNA using the High Capacity cDNA Reverse Transcription Kit (Thermo Fisher Scientific) and then real-time quantitative polymerase reaction (RT-qPCR) analysis was carried out using Fast SYBR™ Green Master Mix (Thermo Fisher Scientific) in triplicate in the LightCycler 480 Real-Time PCR System (Roche Diagnostics, Mannheim, Germany). Glyceraldehyde 3-phosphate dehydrogenase (GAPDH) functioned as the house-keeping gene to normalize the expression of TUG1 and NOTCH1. Previous studies demonstrated that GAPDH could be used for the normalization of target gene expression data [21,22]. The amplification parameters were as follows: denaturation at 95°C for 10 min, followed by 40 cycles of denaturation at 95°C for 30 s, annealing at 60°C for 30 s, and extension at 72°C for 1 min. The primers are listed in Table 1. The 2^−ΔΔCT^ formula was used to examine the gene expression.

The article "Long non-coding RNA TUG1 knockdown hinders the tumorigenesis of multiple myeloma by regulating the microRNA-34a-5p/NOTCH1 signaling pathway" was retracted in 2021. Reason: misconduct by an author.

**Table 1:** Primer sequences

Name	Primer	*T*_m_ (°C)	Product size (bp)	Efficiency (%)
TUG1	F: GCCATGAAGCCCTTTGAG	60	170	97.0
	R: CGGAAGAGTTCAAGGTGTTG			

GAPDH	F: GAAGGTCGGAGTCAACGGATTT	60	226	99.8
	R: CTGGAAGATGGTGATGGGATTTC			

NOTCH1	F: GCCGCCTTTGTGCTTCTGTTC	60	300	98.9
	R: CCGGTGGTCTGTCTGGTCGTC			

U6	F: GCTTCGGCAGCACATATACTAAAAT	60	60	101.6
	R: CGCTTCACGAATTTGCGTGTCAT			

miR-34a-5p	F: CTGGGAGGTGGCAGTGTCTTAGC	60	64	99.3
	R: TCAACTGGTGTCGTGGAGTCGG			

### 2.5 Western blot assay

Total proteins were extracted from the MM cells and xenograft tumors using an ice-cold RIPA lysis buffer (Beyotime, Shanghai, China) containing the protease inhibitor cocktail (Roche Diagnostics) and quantified using the Bio-Rad Bradford Protein Assay Kit (Bio-Rad Laboratories, Hercules, CA, USA). Then, proteins (30 μg per lane) were separated by sodium dodecyl sulfate–polyacrylamide gel electrophoresis and electrotransferred onto nitrocellulose membranes (Millipore, Bedford, MA, USA). After the blockade of nonspecific signals in 5% skimmed milk, the membranes were incubated overnight at 4°C with primary antibodies including anti-GAPDH (1:1,000 dilution; Abcam, Cambridge, UK), anti-NOTCH1 (1:2,000 dilution; Santa Cruz Biotechnology, Dallas, TX, USA), anti-hes family bHLH transcription factor 1 (Hes-1) (1:500 dilution; Abcam), anti-Survivin (Abcam), or anti-Bcl-2 (1:1,000 dilution; Abcam). Next, the membranes were incubated with the corresponding horseradish peroxidase-labeled secondary antibody (1:1,000 dilution; Abcam). Finally, the protein bands were imaged using the Pierce™ ECL Western Blotting Substrate (Thermo Fisher Scientific) in the Bio-Rad ChemiDox XRS imaging system (Bio-Rad Laboratories). Relative quantitative analysis of protein signals was performed by Quantity One software Version 4.1.1 (Bio-Rad Laboratories).

The article "Long non-coding RNA TUG1 knockdown hinders the tumorigenesis of multiple myeloma by regulating the microRNA-34a-5p/NOTCH1 signaling pathway" was retracted in 2021. Reason: misconduct by an author.

### 2.6 Luciferase reporter assay

The binding sites between miR-34a-5p and TUG1 or NOTCH1 were predicted by starBase or TargetScan, respectively. Partial sequences of TUG1 or NOTCH1 3′-UTR containing putative miR-34a-5p complementary sites were sub-cloned into the psiCHECK-2 vector by Hanbio Biotechnology Co., Ltd (Shanghai, China), named as TUG1-Wt or NOTCH1-Wt reporter. Also, TUG1-Mut and NOTCH1-Mut reporter harboring the mutations of miR-34a-5p binding sites were generated by Hanbio Biotechnology Co., Ltd. Then, 400 ng of these constructs and 50 ng of renilla luciferase reporter plasmid (pRL-TK) were, respectively, transfected into NCI-4929 and U266 cells along with miR-NC or miR-34a-5p mimic using Lipofectamine 3000 (Invitrogen, Carlsbad, CA, USA). Forty-eight hours later, luciferase activities were measured by a dual luciferase reporter system (Promega, Madison, WI, USA). Renilla luciferase activities were used as the internal control for the normalization of firefly luciferase activity.

### 2.7 Cell counting Kit-8 assay

The effects of miR-34a-5p and TUG1, alone or in combination, on MM cell proliferation were assessed using the Cell Counting Kit-8 (CCK-8) assay kit (Dojindo Molecular Technologies, Rockville, MD, USA) referring to the protocols of the manufacturer. Briefly, 2 × 10^4^ MM cells in 100 μL of growth medium were plated into 96-well plates. At the indicated time points (0, 24, 48, and 72 h) after transfection, 10 μL of CCK-8 solution was added into each well. After 2 h of incubation, cell absorbance was detected at a wavelength of 450 nm using a microplate reader (BioTek Instruments, Winooski, VT, USA).

### 2.8 RNA pull-down assay

The potential binding ability of TUG1 with miR-34a-5p was tested by the RNA pull-down assay by referring to the protocols described previously [23]. Generally, NCI-4929 and U266 cells were transfected with a biotinylated wild-type TUG1 probe (Bio-TUG1, Sangon Biotech, Shanghai, China), a biotinylated mutant-type TUG1 probe (Bio-TUG1-Mut, Sangon Biotech) harboring the mutations of miR-34a-5p binding sites, or a Bio-NC control probe (Sangon Biotech). At 48 h post transfection, cell lysates were co-incubated with streptavidin-conjugated magnetic beads. The miR-34a-5p levels pulled down by these biotinylated probes were measured by the RT-qPCR assay.

### 2.9 Flow cytometry analysis of cell apoptosis and cell cycle progression

The cell apoptosis pattern was analyzed using the annexin V–FITC Apoptosis Detection Kit (Sigma-Aldrich) by following the protocols of the manufacturer. In general, transfected cells were collected at 48 h after transfection and then resuspended in 1× binding buffer. Next, the cells were stained with annexin V–FITC conjugate and propidium iodide (PI) solution. After 15 min of incubation at room temperature in the dark, cell apoptotic rates were examined by the FACS Calibur flow cytometer (BD Biosciences). For cell cycle analysis, the transfected cells were collected at 48 h post transfection and resuspended in phosphate buffer saline. Then, the cells were fixed with absolute ethanol for 2 h at 4°C and then stained with PI solution for 30 min at 4°C in the dark after the removal of RNA via Rnase A. Finally, the cell distribution patterns in different phases of the cell cycle (G0/G1, S, and G2/M) were detected by flow cytometry (BD Biosciences).

The article "Long non-coding RNA TUG1 knockdown hinders the tumorigenesis of multiple myeloma by regulating the microRNA-34a-5p/NOTCH1 signaling pathway" was retracted in 2021. Reason: misconduct by an author.

### 2.10 Animal experiments

shTUG1 lentiviruses carrying TUG1 knockdown fragment or shNC control lentiviruses were purchased from Hanbio Biotechnology Co., Ltd. For establishment of MM mouse xenograft models, the flanks of male BALB/c nude mice (6 weeks old; Henan Experimental Animal Center, Zhengzhou, China) were subcutaneously inoculated with NCI-H929 cells (5 × 10^6^) infected with shTUG1 or shNC lentiviruses. Tumor volume was measured every 3 days and calculated using the formula: (length × width^2^)/2. On day 30 after injection, the total body weight of mice was measured and xenograft tumors were resected and weighed. The TUG1 and miR-34a-5p levels in xenograft tumors were measured by the RT-qPCR assay. The protein levels of NOTCH1, Hes-1, Survivin, Bcl-2, and GAPDH in xenograft tumors were determined by the Western blot assay.


**Ethical approval:** The research related to animals’ use has been complied with all the relevant national regulations and institutional policies for the care and use of animals. All animal experiments were approved by the Animal Care and Use Committee of Ji’ning No. 1 People’s Hospital and carried out in accordance with the Guide for the Care and Use of Laboratory Animals of the National Research Council.

### 2.11 Statistical analysis

All *in vitro* data obtained from at least three independent experiments are expressed as mean ± standard deviation. The Kaplan–Meier survival analysis was performed. The interaction among TUG1, miR-34a-59, and NOTCH1 was analyzed by Pearson’s correlation analysis. Difference comparisons between groups were performed by Student’s *t*-test, and difference in multiple data was tested by one-way ANOVA along with Tukey’s post hoc test in GraphPad Prism software (La Jolla, CA, USA). Difference with a *P* value below 0.05 was regarded as statistically significant.

The article "Long non-coding RNA TUG1 knockdown hinders the tumorigenesis of multiple myeloma by regulating the microRNA-34a-5p/NOTCH1 signaling pathway" was retracted in 2021. Reason: misconduct by an author.

## 3 Results

### 3.1 TUG1 was highly expressed in MM bone marrow samples and cells

First, the RT-qPCR assay showed that the TUG1 expression was strikingly upregulated in bone marrows of MM patients (*n* = 49) than that in healthy people (*n* = 16) (Figure 1A). Also, a notable upregulation of TUG1 levels was observed in MM cell lines (MM.1S, NCI-H929, and U266) compared with nPCs (Figure 1B). Bone marrow samples of MM patients were divided into the following two groups: high TUG1 expression group (TUG1 level ≥ median value) and low TUG1 expression group (TUG1 < median value) with the median value of TUG1 expression as the cutoff point. The Kaplan–Meier survival analysis revealed that MM patients with high TUG1 expression had a poor survival rate relative to that of the low TUG1 expression group (Figure 1C).

**Figure 1:** TUG1 was highly expressed in bone marrows of MM patients and MM cell lines. (A) TUG1 level was measured by the RT-qPCR assay in bone marrows of MM patients (*n* = 49) and healthy people (*n* = 16). (B) TUG1 level was detected by the RT-qPCR assay in nPCs, MM.1S, NCI-H929, and U266 cells. (C) Kaplan–Meier survival analysis of MM patients according to the difference in TUG1 expression. *P < 0.05.

### 3.2 TUG1 knockdown suppressed cell viability, induced cell cycle arrest and cell apoptosis in MM

Next, three siRNAs targeting TUG1 and a scramble control were synthesized and transfected into MM cells. The transfection efficiency analysis disclosed that these siRNAs targeting TUG1 were efficacious to reduce the TUG1 expression in NCI-H929 and U266 cells (data not shown). To reduce off-target effects, the mixture of these siRNAs targeting TUG1, termed as siTUG1, was used to perform the loss-of-function analysis in MM cells. As shown in Figure 2A, the TUG1 expression level was remarkably downregulated in NCI-H929 and U266 cells following the transfection of siTUG1. Subsequent CCK-8 assay showed that TUG1 knockdown inhibited the cell viability of NCI-H929 and U266 cells (Figure 2B). Moreover, TUG1 loss hampered the cell cycle progression in NCI-H929 and U266 cells, as evidenced by the increase in G0/G1 phase cell proportion and the reduction in S phase cell percentage in siTUG1-transfected cells compared with that of the scramble control group (Figure 2C). In addition, a notable elevation of apoptotic rates was observed in TUG1-depleted NCI-H929 and U266 cells than that in control cells (Figure 2D). These data presented that TUG1 knockdown inhibited cell viability and induced cell cycle arrest and cell apoptosis in MM.

**Figure 2:** TUG1 knockdown suppressed cell proliferation, induced cell cycle arrest and cell apoptosis in MM cells. (A–D) NCI-H929 and U266 cells were transfected with siTUG1 or a scramble siRNA. (A) Forty-eight hours later, the TUG1 level was determined by the RT-qPCR assay. (B) At 0, 24, 48, and 72 h after transfection, the cell viability was assessed by the CCK-8 assay. (C and D) At 48 h post transfection, cell proportions in G0/G1, S, and G2/M phases (C) and cell apoptotic rates (D) were measured by flow cytometry. *P < 0.05.

The article "Long non-coding RNA TUG1 knockdown hinders the tumorigenesis of multiple myeloma by regulating the microRNA-34a-5p/NOTCH1 signaling pathway" was retracted in 2021. Reason: misconduct by an author.

### 3.3 TUG1 negatively regulated the miR-34a-5p expression in MM cells

Bioinformatics prediction analysis by the StarBase database revealed that there existed some complementary bases between TUG1 and miR-34a-5p (Figure 3A), suggesting that TUG1 can interact with miR-34a-5p. Moreover, the RT-qPCR assay manifested that the miR-34a-5p expression was markedly downregulated in the bone marrow samples from MM patients compared with that of the healthy control group (Figure 3B). The TUG1 expression was negatively associated with the miR-34a-5p expression in the bone marrow samples from MM patients (*n* = 49) (Figure 3C). Also, the RT-qPCR assay validated that the introduction of miR-34a-5p mimic could induce the noticeable upregulation of miR-34a-5p levels in NCI-H929 and U266 cells (Figure 3D). Next, the luciferase reporter assay and RNA pull-down assay were performed to further determine whether TUG1 could bind to miR-34a-5p by putative binding sites. The luciferase reporter assay showed that miR-34a-5p mimic triggered the conspicuous downregulation of luciferase activity of the TUG1-Wt reporter covering the predicted miR-34a-5p complementary sites, but had no effect on the luciferase activity of the TUG1-Mut reporter containing mutant miR-34a-5p binding sites in NCI-H929 and U266 cells (Figure 3E and F). The RNA pull-down assay unveiled that miR-34a-5p was enriched by the Bio-TUG1 probe, but not by the Bio-TUG1-mut probe in NCI-H929 and U266 cells (Figure 3G and H). These findings confirmed that TUG1 could bind to miR-34a-5p by putative complementary sites in MM cells. Subsequent RT-qPCR assay presented that silencing of TUG1 promoted the miR-34a-5p expression in NCI-H929 and U266 cells (Figure 3I).

**Figure 3:** TUG1 negatively regulated miR-34a-5p expression in MM cells. (A) Predicted complementary sites between TUG1 and miR-34a-5p by the StarBase database and mutant sites in the TUG1-Mut reporter. (B) The miR-34a-5p level was examined by the RT-qPCR assay in bone marrows of MM patients (*n* = 49) and healthy people (*n* = 16). (C) Correlation analysis between TUG1 and miR-34a-5p in bone marrow samples from MM patients (*n* = 49). (D) The miR-34a-5p level was measured by the RT-qPCR assay at 48 h upon transfection in NCI-H929 and U266 cells transfected with miR-NC or miR-34a-5p mimic. (E and F) NCI-H929 and U266 cells were co-transfected with miR-NC or miR-34a-5p mimic and TUG1-Wt or TUG1-Mut reporter. At 48 h after transfection, luciferase activities were determined by the dual luciferase reporter assay. (G and H) NCI-H929 and U266 cells were transfected with Bio-NC, Bio-TUG1, or Bio-TUG1-mut probe. At 48 h after transfection, the miR-34a-5p level pulled down by the aforementioned biotinylated probes was measured by RNA pull down and RT-qPCR assays. (I) The miR-34a-5p level was measured by the RT-qPCR assay at 48 h after transfection in NCI-H929 and U266 cells transfected with siTUG1 or a scramble siRNA. *P < 0.05.

The article "Long non-coding RNA TUG1 knockdown hinders the tumorigenesis of multiple myeloma by regulating the microRNA-34a-5p/NOTCH1 signaling pathway" was retracted in 2021. Reason: misconduct by an author.

### 3.4 TUG1 functioned as a ceRNA of miR-34a-5p to regulate the NOTCH1 expression in MM cells

TargetScan predicted that NOTCH1 was a potential target of miR-34a-5p (Figure 4A). To further demonstrate this prediction, the effect of miR-34a-5p overexpression on the luciferase activities of the NOTCH1-Wt or NOTCH1-Mut reporter was measured by the luciferase reporter assay. The results displayed that the enforced expression of miR-34a-5p triggered a noticeable decrease in the luciferase activity of the NOTCH1-Wt reporter in NCI-H929 and U266 cells, but no obvious change in the luciferase activity of the NOTCH1-Mut reporter was observed in NCI-H929 and U266 cells after the overexpression of miR-34a-5p compared with that of the miR-NC control group (Figure 4B and C). Moreover, RT-qPCR and Western blot assays presented that TUG1 knockdown or miR-34a-5p increase inhibited the NOTCH1 expression at mRNA and protein levels in NCI-H929 and U266 cells. TUG1 upregulation abrogated the inhibitory effect of miR-34a-5p on NOTCH1 mRNA and protein expression in NCI-H929 and U266 cells (Figure 4D–G). These outcomes manifested that TUG1 could act as a ceRNA of miR-34a-5p to sequester miR-34a-5p from its target NOTCH1, giving rise to the upregulation of NOTCH1 expression in MM cells.

**Figure 4:** TUG1 functioned as a ceRNA of miR-34a-5p to regulate the NOTCH1 expression in MM cells. (A) Putative binding sites between NOTCH1 3′-UTR and miR-34a-5p obtained by TargetScan online website and mutant sites in the NOTCH1-Wt reporter. (B and C) The effect of miR-34a-5p overexpression on luciferase activities of NOTCH1-Wt or NOTCH1-Mut reporter was measured by the luciferase reporter assay at 48 h after transfection in NCI-H929 and U266 cells. (D–G) NCI-H929 and U266 cells were transfected with siTUG1 or its scrambled control, miR-NC, miR-34a-5p mimic, miR-34a-5p mimic + empty vector, and miR-34a-5p mimic + TUG1 overexpression plasmid. After 48 h, NOTCH1 mRNA and protein levels were determined by RT-qPCR and Western blot assays, respectively. *P < 0.05.

The article "Long non-coding RNA TUG1 knockdown hinders the tumorigenesis of multiple myeloma by regulating the microRNA-34a-5p/NOTCH1 signaling pathway" was retracted in 2021. Reason: misconduct by an author.

### 3.5 TUG1 overexpression weakened miR-34a-5p-mediated anti-proliferation and pro-apoptosis effects by regulating the NOTCH1 signaling pathway in MM cells

Next, we further demonstrated that the miR-34a-5p overexpression suppressed cell viability (Figure 5A and B), hindered cell cycle progression (Figure 5C and D) and facilitated cell apoptosis (Figure 5E and F) in NCI-H929 and U266 cells. TUG1 upregulation attenuated the effects of miR-34a-5p on cell proliferation (Figure 5A and B), cell cycle progression (Figure 5C and D) and cell apoptosis (Figure 5E and F) in NCI-H929 and U266 cells. Moreover, overexpression of miR-34a-5p triggered the conspicuous downregulation of Hes-1 (a downstream target of NOTCH1), Survivin (an anti-apoptosis protein), and Bcl-2 (an anti-apoptosis protein) protein levels in NCI-H929 and U266 cells, whereas these effects of miR-34a-5p were weakened by TUG1 increase (Figure 5G and H).

**Figure 5:** TUG1 overexpression weakened miR-34a-5p-mediated anti-proliferation and pro-apoptosis effects by regulating the NOTCH1 signaling pathway in MM cells. (A–H) NCI-H929 and U266 cells were transfected with miR-NC, miR-34a-5p, miR-34a-5p + vector, miR-34a-5p + TUG1 overexpression plasmid. (A and B) Cell viability was evaluated by the CCK-8 assay at 0, 24, 48, or 72 h after transfection. (C–F) Cell cycle distribution pattern (C and D) and cell apoptotic rate (E and F) were measured by flow cytometry at 48 h after transfection. (G and H) Protein levels of Hes-1, Survivin, and Bcl-2 were determined by the Western blot assay at 48 h post transfection. *P < 0.05.

### 3.6 TUG1 knockdown inhibited the growth of MM xenograft tumors by regulating the miR-34a-5p/NOTCH1 signaling pathway

Next, the MM xenograft tumor models were established to explore the effect of TUG1 knockdown on MM tumorigenesis *in vivo.* The results showed that the TUG1 knockdown had no influence on the body weight of mice (Figure 6A). However, TUG1 loss triggered the notable reduction in MM xenograft tumor volume and weight (Figure 6B and C), suggesting that TUG1 deficiency hampered the growth of MM xenograft tumors. Moreover, the RT-qPCR assay further demonstrated that the TUG1 level was remarkably downregulated in MM xenograft tumors infected with shTUG1 lentiviruses (Figure 6D). TUG1 knockdown resulted in the conspicuous increase in miR-34a-5p levels and the marked reduction in the expression of Hes-1, Survivin, and Bcl-2 protein in MM xenograft tumors (Figure 6E and F).

**Figure 6:** TUG1 knockdown inhibited the growth of MM xenograft tumors by regulating the miR-34a-5p/NOTCH1 signaling pathway. (A–F) NCI-H929 cells infected with shTUG1 or shNC lentiviruses were subcutaneously injected into the flanks of mice to establish MM mouse xenograft models with six mice in each group. (A) The total body weight of mice in the shNC and shTUG1 groups was measured on day 30 after injection. (B) Tumor volume was monitored every 3 days for a total of 30 days. (C) Tumors were excised and weighed on day 30 after injection. (D and E) TUG1 and miR-34a-5p levels in xenograft tumors were determined by the RT-qPCR assay. (F) Protein levels of NOTCH1, Hes-1, Survivin, Bcl-2, and GAPDH in xenograft tumors were determined by the Western blot assay. (G) TUG1 promoted MM tumorigenesis by regulating the miR-34a-5p/NOTCH1 signaling pathway *in vitro* and *in vivo*. *P < 0.05.

The article "Long non-coding RNA TUG1 knockdown hinders the tumorigenesis of multiple myeloma by regulating the microRNA-34a-5p/NOTCH1 signaling pathway" was retracted in 2021. Reason: misconduct by an author.

## 4 Discussion

In this study, we demonstrated that TUG1 knockdown inhibited MM cell viability, induced cell cycle arrest and cell apoptosis *in vitro* and hampered MM xenograft tumor growth *in vivo* by regulating the miR-34a-5p/NOTCH1 signaling pathway.

First, we detected the expression patterns of TUG1 in bone marrow samples of MM patients and healthy donors together with MM cells. Our results showed that the TUG1 expression was markedly upregulated in bone marrow of MM patients and in MM cells. Similar results were also obtained in the plasma of MM patients [15]. Moreover, survival analysis revealed that MM patients with high TUG1 expression had a poor prognosis. Functional explorations presented that TUG1 knockdown suppressed MM cell proliferation, blocked cell cycle progression, and promoted cell apoptosis *in vitro*.

Bioinformatics analysis revealed that TUG1 had the possibility to bind with miR-34a-5p. Recently, miR-34a has attracted much attention by virtue of its potential tumor suppressive roles in plenty of malignances by regulating target proteins associated with multiple biological processes such as cell proliferation, cell cycle progression, and cell apoptosis [24,25]. For example, the enforced expression of miR-34a-5p triggered the reduction of cell proliferative, migratory, and invasive abilities and the increase in cell apoptotic activity by silencing Bcl-2 in human cervical carcinoma [26]. The miR-34a-5p overexpression suppressed colorectal carcinoma cell proliferation, migration, and invasion and induced CRC cell apoptosis and cell cycle arrest *in vitro* and hampered CRC xenograft tumor growth *in vivo* [27]. Moreover, the miR-34a overexpression suppressed MM cell proliferation, promoted cell apoptosis and induced cell cycle arrest *in vitro*, and impeded MM xenograft growth *in vivo* [28,29,30]. Xiao et al. pointed out that the miR-34a-5p level was markedly reduced in MM cells and bone marrows of MM patients, and the miR-34a-5p overexpression inhibited proliferation and facilitated apoptosis in MM cells [31]. Furthermore, previous studies showed that TUG1 promoted the development and progression of endometrial carcinoma and hepatoblastoma by regulating miR-34a-5p and downstream targets [32,33]. Consequently, miR-34a-5p was selected as a target of TUG1 to further examine whether TUG1 could exert its function by regulating miR-34a-5p in MM.

The article "Long non-coding RNA TUG1 knockdown hinders the tumorigenesis of multiple myeloma by regulating the microRNA-34a-5p/NOTCH1 signaling pathway" was retracted in 2021. Reason: misconduct by an author.

In this study, we demonstrated that TUG1 could directly bind to miR-34a-5p by bioinformatics analysis, luciferase reporter assay, and RNA pull down assay. TUG1 knockdown triggered the notable upregulation of miR-34a-5p levels in MM cells. Moreover, the miR-34a-5p expression was negatively associated with the TUG1 expression in bone marrow specimens of MM patients. Also, consistent with the previous report [31], the expression of miR-34a-5p was low in bone marrows of MM patients and overexpression of miR-34a-5p suppressed cell proliferation, impeded cell cycle progression, and induced cell apoptosis in MM. Additionally, we further demonstrated that TUG1 upregulation abrogated the effects of miR-34a-5p on cell proliferation, cell cycle progression, and cell apoptosis in MM.

Bioinformatics analysis suggested that NOTCH1 was a potential target of miR-34a-5p. NOTCH1, a transmembrane receptor involved in the regulation of multiple biological processes such as cell growth and cell cycle progression, has been identified as a direct target of miR-34a in glioblastoma multiforme [34], cervical carcinoma, and choriocarcinoma [35]. Moreover, cumulative evidence suggested the key roles of NOTCH1 protein and associated signaling pathways in the onset and progression of multiple carcinomas such as lung carcinoma [36], breast carcinoma [37] and MM [38]. For instance, the enforced expression of NOTCH1 facilitated MM cell proliferation *in vitro* and accelerated MM xenograft tumor growth and angiogenesis *in vivo* [39]. Hence, we further explored whether the TUG1/miR-34a-5p axis could exert its function by regulating NOTCH1 and downstream signaling molecules.

In this study, we further demonstrated that NOTCH1 was a direct target of miR-34a-5p and TUG1 could positively regulate the NOTCH1 expression by miR-34a-5p in MM cells. The Western blot assay disclosed that miR-34a-5p inhibited the expression of Hes-1 (NOTCH1 downstream molecule), Survivin (anti-apoptotic protein), and Bcl-2 (anti-apoptosis protein) in MM cells. Additionally, *in vivo* experiments showed that TUG1 knockdown inhibited MM xenograft tumor growth by upregulating miR-34a-5p and downregulating the expression of NOTCH1, Hes-1, Survivin, and Bcl-2. Consistently, Di Martino et al. revealed that the expression of Bcl-2 and NOTCH1 was markedly downregulated in miR-34a-overexpressed MM cells and xenograft tumors [28].

The article "Long non-coding RNA TUG1 knockdown hinders the tumorigenesis of multiple myeloma by regulating the microRNA-34a-5p/NOTCH1 signaling pathway" was retracted in 2021. Reason: misconduct by an author.

Altogether, our data revealed that TUG1 knockdown inhibited MM tumorigenesis *in vitro* and *in vivo* by regulating the miR-34a-5p/NOTCH1 signaling pathway. To our knowledge, this study was first to elucidate the roles and molecular basis of TUG1 in MM tumorigenesis, providing some potential biomarkers for MM diagnosis and prognosis, and possible targets for the treatment of MM. However, the effects of TUG1/miR-34a-5p/NOTCH1 axis on MM tumorigenesis need to be further validated by more experimental approaches in other MM cell lines and xenograft models.
